# Pricing Israeli Option with Time-changed Compensation by an FFT-Based High-order Multinomial Tree in Lévy Markets

**DOI:** 10.1155/2022/9682292

**Published:** 2022-06-29

**Authors:** Weiwei Wang, Xiaoping Hu

**Affiliations:** ^1^School of Applied Technology, Nanjing University of Information Science and Technology, Nanjing 210044, China; ^2^School of Economics and Management, Southeast University, Nanjing 210096, China

## Abstract

The problem for pricing the Israel option with time-changed compensation was studied based on the high-order recombined multinomial tree by using a fast Fourier transform to approximate a Lévy process. First, the Lévy option pricing model and Fourier transform are introduced. Then, a network model based on FFT (Markov chain) is presented. After that, an FFT-based multinomial tree construction method is given to solve the problem of difficult parameter estimation when approximating the Lévy process with high-order multinomial trees. It is proved that the discrete random variables corresponding to the multinomial tree converge to the Lévy-distributed continuous random variable. Next, an algorithm based on a reverse recursion algorithm for pricing the Israel option with time-changed compensation was presented. Finally, an example was illustrated, and the relationship between the price of the Israel option and the time-changed compensation was discussed. The results show that the method of constructing a high-order recombined multinomial tree based on FFT has very high calculation precision and calculation speed, which can solve the problem of traditional risk-neutral multinomial tree construction, and it is a promising pricing method for pricing Israel options.

## 1. Introduction

Israel option is a game option, and pricing the Israel option is a very difficult problem (a reference to Roux [1]). Both Dumitrescu et al. [2] and Essaky and Hassani [3] studied the pricing problem of the Israel option based on the BSDE method. Dolinsky and Kifer [4] investigated the risk minimization issue of the Israel option with transaction costs. Ekström et al. [5] gave a method for pricing the Israel option while there were heterogeneous beliefs in the market. In recent years, the Fourier transform has been widely applicated to pricing derivatives. On one hand, because of the implementation of a fast Fourier transform, the computational complexity can be reduced from *N*^2^ to *N*log_2_^*N*^, which greatly improves the computational efficiency. On the other hand, the Lévy process can better describe the phenomenon of “excess kurtosis, fat tail, and negative skewness” of the underlying assets, while the Lévy process does exist as an analytic form of the characteristic function. The majority of the Lévy process does not exist an analytic form of the density function. Based on the Fourier transform, Fang and Oosterlee [6], Dia [7], Kwok et al. [8], Zhang and Wang [9], Ortiz-Gracia and Oosterlee [10] studied the European option pricing problem when the underlying asset was described by the Lévy process. Eberlein [11] systematically introduced various methods of Fourier transform pricing for European options. Dempster and Hong [12], Pellegrino and Sabino [13], and Andersson [14] discussed the spread options pricing problem based on Fourier transform. Ramponi [15] under the condition of jump diffuse of the underlying asset price obedience mechanism, the Fourier transform method of pricing the forward start option is given. Zhang and Oosterlee [16] introduced the pricing of the American Asian option under the Lévy model by using Fourier cosine expansion. Ibrahim et al. [17] gave the Fourier transform method for pricing extendable options (extendible options) method, and Fusai [18], Shu [19], and Huang et al. [20] used the Fourier method to study the pricing problem of the different forms of Asian options. Fang and Oosterlee [21] and Eberlein et al. [22]discussed the pricing problem of barrier options and exotic options under Fourier transform. Mordecki [23], Sheu and Tsai [24], Yamazaki [25], Boyarchenko, and Levendorskii [26] showed the optimal stochastic and long-term American option pricing problem by taking Fourier transforms. Based on the Fourier transform, Zhylyevskyy [27], Gyulov, and Valkov [28] generalized the pricing of American options on stochastic volatility and finite interval. Pellegrino and Sabino [13], Ruijter and Oosterlee [29], and Chan [30] took multidimensional Fourier transform to derive option pricing. Given FFT, a Markov chain is used for option pricing by Wong and Guan [31]. In Madan and Yor [32], the expression theorem of time-varying Brownian for a class of Lévy processes was given. The risk pricing under the Lévy process is given in Asiimwe et al. [33]. Kulczycki and Ryznar [34] focused on the Lévy process transfer probability estimation problem. Neufeld and Nutz [35] studied the characteristic functions of nonlinear Lévy processes. And the characteristic function of the time-inhomogeneous Lévy-driven O–U process is given in Vrins [36]. Zeng and Kwok [37] developed the pricing and approximation of arithmetic average Asian options under the time-varying Lévy process. The Lévy model in Jovan and Ahčan [38] is applied to the problem of default prediction using structured methods. Gong and Zhuang [39], and Lian et al. [40] studied the pricing methods of American options and discrete barrier options under the Lévy process, respectively.

In the existing literature, the authors focus on pricing the Israel option with constant compensation. However, in practice, there exists a type of Israel option with time-changed compensation (Zaevski [41]). The method of approximating the Lévy process is proposed based on a fast Fourier transform and an algorithm for pricing the Israel option with time-changed compensation. The Fourier transform itself has high computational efficiency; however, the existing Fourier transform method for calculating derivatives prices requires massive unnecessary calculations, such as the need to calculate the price of options under different strike prices, whether the strike price is needed, and whether the market exists, resulting in wasted computational resources and inefficient computation. The Markov chain method has too many nodes at the beginning of the computation and a fixed number of nodes at the end of the computation. Therefore, the same computational efficiency is not high. This paper gives a method to construct a multinomial tree to approximate the Lévy process based on FFT, which can effectively solve the parameter estimation problem in multinomial tree construction.

The rest of this paper is organized as follows: Section 2 introduces the Lévy model, for option pricing, and Fourier transform.  Section 3 describes the FFT-based network.  Section 4 gives a method to construct a recombined multinomial tree via FFT. In section 5, an algorithm for pricing the Israel option is given. In section 6, an example is illustrated.  Section 7 is conclusions.

## 2. Lévy Option Pricing and Fourier Transform

The Lévy process is an independent and steady increment process, and each Lévy process corresponds to an infinitely separable distribution. Denote *X*_*t*_ as a Lévy process. According to Lévy–Khintchine formula, the characteristic exponent of *X*_1_ is

(1) $$\begin{array}{c} \Psi \left(u\right)=i\mu u-\frac{1}{2}\sigma^{2}u^{2}+\int_{\mathbb{R}}\left(e^{iux}-1-iux1_{\left(-1,1\right)}\right)\nu \left(\text{d}x\right). \end{array}$$

The characteristic function *X*_*t*_ is

(2) $$\begin{array}{c} \Phi \left(u\right)=E_{X_{t}}\left[e^{iux}\right]=e^{t\Psi \left(u\right)}. \end{array}$$

Wong and Guan [31] showed several characteristic functions of the Lévy process which are commonly used in the pricing of financial derivatives. In addition to the Wiener process, most of the commonly used Lévy process only has an analytical form of the characteristic function, and there is no analytical form of probability density function(PDF) *f*(*x*) or cumulative distribution function (CDF) *F*(*x*).

The characteristic function is the Fourier transform of the probability density function, as follows:

Φ(*u*)=∫_−*∞*_^+*∞*^*e*^*iux*^*f*(*x*)d*x*.

By using the inverse Fourier transform, the probability density function and the cumulative distribution function can be obtained from the characteristic function.

(3) $$\begin{array}{c} f\left(x\right)=\frac{1}{\pi }\int_{0}^{+\infty }ℜ\left(e^{-ixu}\Phi \left(u\right)\right)\text{d}u,\\ F\left(x\right)=\frac{1}{2}-\frac{1}{\pi }\int_{0}^{+\infty }J\left(\frac{e^{-ixu}\Phi \left(u\right)}{u}\right)\text{d}u. \end{array}$$

ℜ(.) is the real part of the complex number, and *𝔍*(.) is the imaginary part of the complex number. Under the risk-neutral probability measure, the price of the European option with the maturity *T* and the value of payment function *g*(.) at *t*=0 is

(4) $$\begin{array}{c} C=e^{-rT}E^{Q}\left[g\left(x\right)\right]\\ =e^{-rT}\int_{-\infty }^{+\infty }g\left(x\right)f\left(x\right)\text{d}x. \end{array}$$

Theoretically, the probability density function can be obtained from equation (3), and the value of the option can be calculated by equation (4). However, we cannot obtain the analytical form of the probability density function for most Lévy processes unless the numerical method is used, which is extremely inefficient. Carr and Madan [42] and Lewis [43] changed the strike price of the European call option and introduced an exponential damping factor into the payoff function. After that, option pricing was transformed into the inner product of Fourier space by Plancherel–Parseval's theorem. Based on the discounted cumulative distribution function, the analytic pricing formula of the Fourier transform space is obtained in Bates [44].

Even if the European option pricing formula is obtained in the Fourier space, it is necessary to use the inverse Fourier to get the true European option price. There is no analytic form pricing formula in Fourier space for path-dependent exotic options, and American options can be executed ahead of time. When we compute the Fourier transform or the inverse Fourier transform by a numerical method, FFT (IFFT) uses the symmetry and periodicity of a complex number to simplify the calculation of *N*^2^ times which is necessary for calculating discrete Fourier transform or inverse Fourier transform to *N*log_2_^*N*^ times. In derivatives pricing, if we can get the analytic pricing formula of Fourier space, it is also known as the analytic pricing formula.

## 3. FFT-Based Networks

For the path-dependent option under the Lévy model, Wong and Guan [31] presented a method of building a network model using FFT, which is essentially a discrete-time finite-state Markov chain. In the network model of Wong and Guan [31], the time is evenly discretized. In each period, the number of nodes in the network is fixed. Each node is connected to all the nodes in the next period. The network structure is shown in Figure 1.

When the probability transfer matrix is calculated, the conditional density function *f*(*x*_*j*_) at the *N*-equidistant node is calculated by FFT using the conditional feature Φ(*u*|*x*_*i*_) of *x*_*i*_ at the *i*-th node, and the transition probability is calculated as follows:

(5) $$\begin{array}{c} P_{ij}\left(t\right)=\frac{f\left(x_{j}|x_{i}\right)}{\sum_{k=1}^{N}f\left(x_{k}|x_{i}\right)}. \end{array}$$

In the above formula, the denominator is an approximate probability density function in a finite interval, and there exists a truncation error. The denominator can be seen as a solution to ensure that the transition probability matrix satisfies the sum of the row elements is 1. Based on the network model, Wong and Guan [31] described the pricing method for the European option and American option. Combining forward shot grids (FSGs), we also give pricing methods for the Asian option and the lookback option.

The network model is applied to the pricing of derivatives. In the whole calculation process, the nodes remain fixed, and the computation is controllable. However, in the initial stage, the price movement of the underlying asset is concentrated near the initial price. The excessively large calculation interval and the number of computing nodes cannot significantly affect the calculation accuracy, resulting in the waste of computing resources. Near maturity, the underlying asset price fluctuates greatly. This region has a significant influence on the derivative price (especially for the European option). It requires a larger calculation interval and more computing nodes. Besides, when calculating the transition probability matrix, it is necessary to use the conditional characteristic function of the Lévy process. These factors lead to the inefficiency of the network method when calculating the derivative price.

## 4. FFT-Based Recombined Multinomial Trees

The recombined multinomial tree uses the node recombination technology to realize that the node number grows linearly with the number of periods and overcomes the shortcomings of the general multinomial tree nodes growing exponentially with the number of periods. It is very difficult to determine parameters to meet conditions in the multinomial tree. It is often necessary to add some extra constraints, such as Yamada and Primbs [45] established penta-nominal tree parameter estimation formulation and required that the kurtosis and skewness of the continuous distribution must satisfy certain conditional relations, which limits the use scope of recombined multinomial tree. Moreover, it is because of the limitation of the moment matching technique that there is no multinomial tree with more than 5 states. Hu [46] used the saddle-point approximation method to construct the construction method for the multinomial tree approximation Lévy process. The advantage of the saddle-point approximation is that the computation is fast; however, the computation interval of interest cannot be selected, and the accuracy of the approximation cannot be changed.

The underlying asset price follows the exponential Lévy process under the risk-neutral probability measure.

(6) $$\begin{array}{c} S_{t}=S_{0}e^{\left(rt-\mu t+X_{t}\right)}, \end{array}$$

where *S*_0_ is the stock price at *t*=0, *r* > 0 is the risk-free interest rate, *X*_*t*_ follows the Lévy process, *μ* is the constant that makes the expected return rate on assets in equation (6) equal to the risk-free rate. *T* > 0 is maturity, *δ*=*T*/*N*. Due to the properties of independent stationary increment of the Lévy process, we have

(7) $$\begin{array}{c} \log\left(S_{n\delta }\right)-\log\left(S_{\left(n-1\right)\delta }\right)=\left(r-\mu \right)\delta +X_{\delta }. \end{array}$$

Without citing confusion, we denote *S*_*n*_ : =*S*_*nδ*_, *X*_*n*_ : =*X*_*nδ*_ and *X*_*δ*_ as approximation Lévy distribution in [0, *δ*] of *L*=2^*k*^ state multinomial tree. The truncation interval *X*_*δ*_ is [−*a*, *a*]. Given Δ=2*a*/*L* − 1, that we have

(8) $$\begin{array}{c} x_{1,j}=-a+\Delta j,\\ j=0,1,2,\ldots ,L-1. \end{array}$$

There are (*L* − 1)*n*+1 nodes in the phase *n*(*n* ≤ *N*) of *L*-state recombined multinomial tree. And, the *j*-th node follows

(9) $$\begin{array}{c} x_{n,j}=-na+\Delta j,\\ j=0,1,2,\ldots ,\left(L-1\right)n. \end{array}$$

In the *n*-th period, the truncation interval of *X*_*n*_ is [−*na*, *na*]. Considering

(10) $$\begin{array}{c} X_{n+1,j+k}=-\left(n+1\right)a+\left(j+k\right)\Delta ,\\ =-na+j\Delta -a+k\Delta ,\\ =X_{n,j}+X_{1,k}, \end{array}$$

where *k*=0,1,2,…, *L* − 1 . Thus, we denote *X*_*n*+1,*j*_,…, *X*_*n*+1,*j*+*L*−1_ as the *L*-th node in the *n*+1 th period from *n*-th node in the period *n*. The price of the underlying asset at the *j* th node in the period *n* is

(11) $$\begin{array}{c} S_{n,j}=S_{0}e^{\left(\left(r-\mu \right)\delta n+X_{n,j}\right)}\\ =S_{0}e^{\left(\left(r-\mu \right)\delta n-na+j\Delta \right)},\;j=0,1,2,\ldots ,\left(L-1\right)n. \end{array}$$

Φ(*u*) is a characteristic function in [0, *δ*] of the Lévy process. And the probability density function (3) is discretized as

(12) $$\begin{array}{c} f\left(x\right)=\frac{1}{\pi }\int_{0}^{+\infty }ℜ\left(e^{-ixu}\Phi \left(u\right)\right)\text{d}u\approx \frac{1}{\pi }\sum_{j=0}^{L-1}ℜ\left(e^{-ixu_{j}}\Phi \left(u_{j}\right)\right)\eta . \end{array}$$

The upper bound of the integral (12) is *b*=*Lη*, with Δ*η*=2*π*/*L*, so that the FFT can be used to calculate the equation (12). Values of *x* can be obtained with the use of FFT. Given

(13) $$\begin{array}{c} x_{j}=-a+\Delta j,\;j=0,1,2,\ldots ,L-1. \end{array}$$

*x*_*j*_ ∈ [−*a*, *a*]. Let *u*_*j*_=*ηj* further then equation (12) can be expressed as

(14) $$\begin{array}{c} f\left(x_{k}\right)\approx \frac{1}{\pi }\sum_{j=0}^{L-1}ℜ\left(e^{-i\Delta \eta kj}\Phi \left(u_{j}\right)\eta w_{j}\right), \end{array}$$

where *k*=0,1,2,…, *L* − 1, *w*_*j*_ is the weight coefficient based on different numerical integration methods, for example, the regular weight coefficient of the Trapezoidal rule *w*_*j*_=1/2, when *j*=0, *L* − 1, otherwise *w*_*j*=1_, the weight coefficient of Simpson's rule based on cubic polynomial is

(15) $$\begin{array}{c} \;w_{j}=\left\{\begin{array}{c} \frac{1}{3},\;j=0,L-1,\\ \frac{4}{3},\;j=1,3,5,\ldots ,L-3,\\ \frac{2}{3},\;j=2,4,6,\ldots ,L-2. \end{array}\right. \end{array}$$

Using FFT, we can get the approximate value of the probability density function at the inner-equidistant grid point [−*a*, *a*].

The probability of occurrence of a state *j* in a state tree *L* is

(16) $$\begin{array}{c} P_{j}=\frac{f\left(x_{j}\right)}{\sum_{k=0}^{L-1}f\left(x_{k}\right)}. \end{array}$$

The denominator in (16) guarantees that all states in the multinomial tree *L* can form a complete probability space.

**Theorem 1 .**

When *a*⟶+*∞*, *L*⟶+*∞*, discrete random variables *X*_1,*j*_ converge in distribution continuous distribution *X*_*δ*_.

**Proof**

The density function of *X*_*δ*_ is *f*(*x*),  *x* ∈ (−*∞*, +*∞*), *X*_1,*j*_ represents the *L* aliquot grid points within [−*a*, *a*], we can extend the discrete random variables *X*_1,*j*_ to be continuous distribution in [−*a*, *a*], and the cumulative distribution function is

(17) $$\begin{array}{c} \tilde{F}\left(x\right)=\left\{\begin{array}{c} P_{0},\;x\leq -a,\\ \sum_{k=0}^{j}P_{k},\;-a+\Delta j<x\leq -a+\Delta \left(j+1\right),\\ 1,\;x>a. \end{array}\right. \end{array}$$

- If *x* ≤ −*a* , because of monotonically increasing property of *F*(*x*), we have $\left|F\left(x\right)-\tilde{F}\left(x\right)\right|\leq F\left(x\right)+\tilde{F}\left(x\right)\leq F\left(-a\right)+\tilde{F}\left(-a\right)\leq F\left(-a\right)+f\left(-a\right)$
- ∵lim_−*a*⟶−*∞*_*F*(−*a*)=lim_−*a*⟶−*∞*_*f*(−*a*)=0
- ∴$\lim_{-a⟶-\infty x\leq -a}\left|F\left(x\right)-\tilde{F}\left(x\right)\right|=0$
- If *x* ≥ *a*, we have $\left|F\left(x\right)-\tilde{F}\left(x\right)\right|=\left|F\left(x\right)-1\right|$
- ∵lim_*a*⟶+*∞*_*F*(*a*)=1
- ∴$\underset{\begin{array}{c} a⟶+\infty \\ x\geq a \end{array}}{\lim}\left|F\left(x\right)-\tilde{F}\left(x\right)\right|=0$
- If −*a*+Δ*j* < *x* ≤ −*a*+Δ(*j*+1), *j*=1,2,…, *L* − 1, we have
- $\begin{array}{c} \tilde{F}\left(x\right)=\sum_{k=0}^{j}P_{k}\\ =\sum_{k=0}^{j}f\left(x_{k}\right)/\sum_{i=0}^{L-1}f\left(x_{i}\right)\\ =\sum_{k=0}^{j}f\left(x_{k}\right)\Delta /\sum_{i=0}^{L-1}f\left(x_{i}\right)\Delta \end{array}$
- ∵the *a* is fixed, *L*⟶+*∞* , Δ=2*a*/*L* − 1⟶0 , *x*_*j*_⟶*x*
- ∴ $\lim_{L⟶+\infty }\tilde{F}\left(x\right)=F\left(x\right)-F\left(-a\right)/F\left(a\right)-F\left(-a\right)$
- ∵When *a*⟶+*∞*, *F*(−*a*)⟶0, *F*(*a*)⟶1
- ∴ $\lim_{a⟶+\infty }\lim_{L⟶+\infty }\tilde{F}\left(x\right)=F\left(x\right)$
- Integrated (i), (ii) and (iii), ∀*x* ∈ (−*∞*, +*∞*) , we have
- $\underset{\begin{array}{c} L⟶+\infty \\ a⟶+\infty \end{array}}{\lim}\tilde{F}\left(x\right)=F\left(x\right)$

That is, the distribution of the discrete random variable *X*_1,*j*_ converges to the continuous distribution *X*_*δ*_.

## 5. Pricing Israel Options

Israel or game options are first introduced by Kifer [47]. The Israel option is the contract between the writer and the holder, and both have the right to exercise at any stop time before the expiry date. If the holder exercises in time, he or she receives the number *y*_*t*_ from the writer, if the writer cancels the contract before the holder, he must pay *x*_*t*_ ≥ *y*_*t*_ to the holder, so that *x*_*t*_ − *y*_*t*_ is deemed to be a penalty for the cancellation of the contract. If the writer and the holder exercise the contract at the same time, the holder receives y_*t*_, which is the value received by the holder for the early exercise of the option.

(18) $$\begin{array}{c} {\text{Let}}^{1}y_{t}={\left(K-S_{t}\right)}^{+}. \end{array}$$

where *x^+^* = max (*x*, 0) and *x*_*t*_=*y*_*t*_+*η*_*t*_, is the payment received by the option holder when the option is cancelled by the option issuer, where *η*_*t*_ is the additional compensation paid by the option issuer when the option is cancelled and is a deterministic function of time. For example, *η*_*t*_ is described as follows:

(19) $$\begin{array}{c} \eta =\eta \left(t\right)\\ =\alpha e^{\beta \left(T-t\right)}, \end{array}$$

where *α* > 0, *β* ≥ 0.

*β* > 0 indicates that the earlier the seller cancels the contract, the more compensation is needed. If *α* is very large, the Israel option degenerates into an American option.

The time step is *δ* in the recombined multinomial tree with *L* states, let *η*_*n*_=*αe*^*β*(*N* − *n*)*δ*^, and *v*_*n*,*j*_ is the price of Israel option at the *n* − *th* period *j* − *th* node, and *c*_*n*,*j*_ is the continued value at this node. According to the risk-neutral pricing method, the price of the Israel option is obtained by

(20) $$\begin{array}{c} v_{n,j}=\min\left(x_{n,j},\max\left(y_{n,j},c_{n,j}\right)\right), \end{array}$$

where

(21) $$\begin{array}{c} c_{n,j}=e^{-r\delta }\sum_{k=0}^{L-1}p_{i}v_{n+1,j+k}. \end{array}$$

At the mature time *t*=*T*, *v*_*N*,*j*_=*y*_*N*,*j*_, and *c*_*N*,*j*_=0, *j*=0,…, (*L* − 1)*N*. And at the initial time *t*=0, the price of the Israel option *p* is equal to *p*=*v*_0,0_=*c*_0,0_.^1^(*x*)^+^=max(0, *x*)

## 6. Illustration

Lévy distribution must have a characteristic function but not a probability distribution function in analytical form. The Lévy process is widely used in the random process of financial modeling. For example, Carr et al. [48] pointed out that the CGMY process is a pure bouncing random Lévy process that does not contain continuous Brownian motion. Within the appropriate scope of the parameter, the CGMY process can guarantee an infinite number of bouncing at any finite time interval. The price movements of risky assets constitute infinitely many small jumping and a small number of large jumping. It is more close to the actual financial market. The characteristics function of CGMY distribution is

(22) $$\begin{array}{c} \Phi \left(\mu \right)=e^{C\Gamma \left(-Y\right)\left({\left(G+i\mu \right)}^{Y}-G^{Y}+{\left(M-i\mu \right)}^{Y}-M^{Y}\right)}. \end{array}$$

Γ(.) is the Gamma function, *C*, *G*, *M*, *Y* is the parameter of CGMY distribution, *C*, *G*, *M* > 0, *Y* < 2. However, if 1 ≤ *Y* < 2, there is no limited second moment; if 0 ≤ *Y* < 1, the corresponding CGMY process has infinitely many bouncing. For the CGMY process, there are

(23) $$\begin{array}{c} M_{\text{saddle}}\left(u\right)=C\Gamma \left(-Y\right)\left({\left(G+iu\right)}^{Y}-G^{Y}+{\left(M-iu\right)}^{Y}-M^{Y}\right), \end{array}$$

due to

(24) $$\begin{array}{c} M_{\text{saddle}}^{\left(j\right)}\left(u\right)=i^{j}C\Gamma \left(j-Y\right)\left({\left(G+iu\right)}^{Y-j}+{\left(-1\right)}^{j}{\left(M-iu\right)}^{Y-j}\right),\;j=1,2,3,4,\ldots . \end{array}$$

According to equation (6), that is,

(25) $$\begin{array}{c} {\left(G+\alpha_{s}^{*}\right)}^{Y-1}-{\left(M-\alpha_{s}^{*}\right)}^{Y-1}=\frac{x}{C\Gamma \left(1-Y\right)}. \end{array}$$

Taking infinite bouncing of the CGMY process into consideration, that is, 0 ≤ *Y* < 1, the left of equation (25) is continuous and monotone decreasing at the interval (−*G*, *M*), the value range is (−*∞*, +*∞*). So for arbitrary *x*, there will be a unique solution at the interval (−*G*, *M*).

Geman [49] estimated stock price based on data of PJM company, *σ*_0_=20%, skewness is *s*_0_=−0.98, kurtosis is *κ*_0_=15.11, parameters of CGMY distribution are *C*=0.279627, *G*=1.497869, *M*=1.97856, *Y*=0.257689. *T*=0.5, the annual risk-free interest rate is *r*=5%, the initial stock price is *S*_0_=100, the strike price is *K*=80 : 1 : 120, the number of states is *L*=1024, multinomial trees period *N*=50. Let *α*=5, *β*=±0.5, 0 in the equation (19).

From Figure 2, the fact that the price of the Israel option increases with the increase *β* can be easily discovered, which is consistent with the fact that equation (2) is a decrement function of *β*. Furthermore, the change of *β* has a significant effect on the Israel option price while the strike price is near to the initial time price of the stock, and the effect on the prices of both the deep-out-of-money Israel option and the deep-in-the-money Israel option is not significant. The time-varying compensated Israeli option degenerates into an ordinary Israeli option when *β*=0.

## 7. Conclusion

In this paper, we use the characteristic function of the Lévy process to obtain the function value of the probability density function in a given interval and directly use the probability density function value at these lattice points to generate the risk-neutral probability. It is proved that the discrete random variables corresponding to the multinomial tree converge to the Lévy distribution of a continuous random variable. Compared with binary trees, multinomial trees have more number of states and thus have faster convergence when the number of periods is the same. The algorithm for pricing the Israel option with time-changed compensation was obtained, and the relationship between the price of the Israel option and *β* was also discussed.

Although the recombined multinomial tree improves computational efficiency in the period of underlying asset price fluctuating slightly, however, with the increase of the number of multinomial tree periods, the number of nodes increases linearly, and the computation interval of the FFT recombined multinomial tree also increases linearly. To recombine the multinomial tree, the calculation interval of each option multinomial tree is the same, and sometimes, it will lead to the calculation interval being too large and reduce the calculation efficiency. In the whole process of the Markov chain, the number of nodes remains unchanged, so the efficiency of the Markov chain is low in the period when the price of the underlying asset fluctuates a little. Therefore, the Lévy model of the option pricing method based on the FFT, combined with the respective advantages of recombined multinomial lattices and Markov chains, will be studied in the future. In addition, according to our research, the multinomial tree method, like the binomial tree method, has the so-called numerical instability and numerical oscillation phenomena, and we will continue to study the methods and means to suppress the numerical instability and numerical oscillation of multinomial trees in the future.

## Figures and Tables

**Figure 1:** FFT-network models.

**Figure 2:** Prices of Israel options with different strike prices.

## Data Availability

All data used in this paper can be reached by request to the authors.
